The article "Rhubarb Enema Increasing Short-Chain Fatty Acids that Improves the Intestinal Barrier Disruption in CKD May Be Related to the Regulation of Gut Dysbiosis" was published in 2022. Journal: Biomed Res Int.

# Rhubarb Enema Increasing Short-Chain Fatty Acids that Improves the Intestinal Barrier Disruption in CKD May Be Related to the Regulation of Gut Dysbiosis

**DOI:** 10.1155/2022/1896781

**Published:** 2022-01-20

**Authors:** Chunlan Ji, Fuhua Lu, Yuchi Wu, Zhaoyu Lu, Yenan Mo, Lijuan Han, Qizhan Lin, Xusheng Liu, Chuan Zou

**Affiliations:** ^1^Second Clinical Medical College, Guangzhou University of Chinese Medicine, Guangzhou 510405, China; ^2^Department of Nephrology, Guangdong Provincial Hospital of Chinese Medicine, Guangzhou 510120, China; ^3^State Key Laboratory of Dampness Syndrome of Chinese Medicine, The Second Affiliated Hospital of Guangzhou University of Chinese Medicine, Guangzhou 510120, China; ^4^Department of Bioinformatics, Guangdong Provincial Hospital of Chinese Medicine, Guangzhou 510120, China

## Abstract

The incidence of CKD seriously endangers people's health. Researchers have proposed that improving the intestinal barrier damage in CKD may be an effective target for delaying the progression of CKD. Rhubarb can effectively improve the intestinal barrier and renal fibrosis, which may be related to the regulation of gut dysbiosis, but the mechanism needs to be further studied. Short-chain fatty acids (SCFAs) are important metabolites of the gut microbiota and play an important role in maintaining the intestinal barrier. The purpose of this study was to investigate whether rhubarb enema regulates the production of short-chain fatty acid-related gut microbiota and improves the intestinal barrier damage of CKD. 5/6 nephrectomy rats were used as the animal model, sevelamer was used as the positive control group, and the sham operation rats were used as the control group. After 4 weeks of enema treatment, the general clinical indicators, short-chain fatty acid levels, renal pathology, intestinal tissue pathology, intestinal tight junction protein, and changes in gut microbiota were detected. The results showed that rhubarb enema can increase the level of short-chain fatty acids in the 5/6 nephrectomy model rats, improve the intestinal barrier damage, inhibit the decrease of intestinal tight junction proteins, reduce inflammation levels, improve kidney pathology, reduce blood creatinine levels, and regulate the intestinal tract, the abundance, and composition of the flora. Further correlation analysis showed that rhubarb enema increased the level of short-chain fatty acids in 5/6 nephrectomy model rats, which may be related to the 7 strains that may regulate the production of short-chain fatty acids. This study indicated that rhubarb enema can improve the intestinal barrier damage of 5/6 nephrectomy model rats and improve CKD, which may be related to the regulation of short-chain fatty acid-producing gut microbiota.

The article "Rhubarb Enema Increasing Short-Chain Fatty Acids that Improves the Intestinal Barrier Disruption in CKD May Be Related to the Regulation of Gut Dysbiosis" was published in 2022. Journal: Biomed Res Int.

## 1. Introduction

Chronic kidney disease (CKD) is a disease in which the development of chronic kidney structural damage and dysfunction caused by various reasons can lead to chronic renal failure (CRF). Currently, more than 850 million people in the world suffer from chronic kidney disease, of which 5–10 million are end-stage patients [1], which seriously endangers people's lives and health. Therefore, the international nephrology communities have been committed to exploring the risk factors of CKD progression and new methods to alleviate the progression of CKD.

Recent studies have found that in the state of CKD, the disorder of the intestinal flora produces a variety of metabolic toxins, which enter the circulation through the injured intestinal barrier to promote cardiovascular and kidney damage [2], further aggravating the progression of CKD and is closely related to poor clinical prognosis [3]. Based on these connections between the intestine and the kidney, the “gut-kidney axis” theory has been formed [4]. It has become the focus of research in nephrology circles in recent years. The intestinal barrier is one of the key links in this theory, and there is still a lack of research on the treatment of CKD intestinal barrier injury.

Short-chain fatty acids (SCFAs) are also called volatile fatty acids. According to the number of carbon atoms in the carbon chain of organic fatty acids, organic fatty acids with carbon atoms of 1-6 are called SCFAs, which mainly include acetic acid, propionic acid, isobutyric acid, butyric acid, isovaleric acid, valeric acid, and hexanoic acid. SCFAs are mainly derived from intestinal bacteria, such as *akkermansia*, *muciniphila*, *bacteroides* spp., *bifidobacterium* spp., *prevotella* spp., and *ruminococcus* spp., which are produced by decomposing ingested dietary fiber [5]. SCFAs provide 60-70% of the energy source for intestinal epithelial cells [6]. In addition, SCFAs can regulate intestinal immune cells to produce IL-22, regulate Th1 cells to produce IL-10, regulate intestinal immunity, and protect the intestinal mucosa [7, 8].

The intestinal mucosa is an important barrier to prevent pathogenic microorganisms in the intestinal cavity from entering the circulation [9]. The CKD intestinal barrier is affected by various urinary toxins accumulated in the intestinal cavity; for example, uremia plasma depletes the tight junction protein component of the intestinal epithelium and impairs the barrier function [10]. The injury of the intestinal barrier in CKD provides a prerequisite for the translocation of intestinal bacteria to the submucosa and CKD-associated inflammation, which may be related to the dysbiosis and the decrease of SCFAs [11, 12]. Studies found that the abundance of CKD intestinal flora was significantly changed, and the content of SCFAs in CKD intestinal tract decreased significantly, especially butyrate, which were closely related to the progress of CKD [13]. Therefore, regulating the dysbiosis and increasing the content of SCFAS may be a potential target to improve the intestinal barrier damage and delay the progression of CKD.

The article "Rhubarb Enema Increasing Short-Chain Fatty Acids that Improves the Intestinal Barrier Disruption in CKD May Be Related to the Regulation of Gut Dysbiosis" was published in 2022. Journal: Biomed Res Int.

In addition, CKD brings heavy pill burden. A mean of 9-13 medications per day in advanced CKD patients was reported [14]. Enema with medical solutions administered via an anal catheter avoids increasing the burden. Retention enema with rhubarb-based formula decoction has been applied to treat chronic kidney failure since 1950s in China. Rhubarb has been used to treat chronic renal failure for a long history. Rhubarb comprises the dried roots and rhizomes of rheum palmatum L (http://www.theplantlist.org/). Evidence is accumulating for rhubarb enema in treatment of CKD [15–18], but its mechanism of action has yet to be revealed.

We have conducted a series of studies on the related mechanisms of rhubarb enema delaying the progression of CKD. We found that rhubarb enema can significantly reduce the level of oxidative stress and systemic inflammation in CKD rats and improve renal interstitial fibrosis [19]. With the introduction of the intestinal-renal axis theory, our further research found that rhubarb enema can reduce intestinal-derived LPS and downregulate the intestinal mucosal immune inflammation mediated by the LPS-TLR4 signaling pathway, thereby improving the intestinal barrier damage and improving the inflammation of the CKD system and renal fibrosis. Moreover, the improvement of intestinal mucosal inflammation by enema may be related to the regulation of related intestinal bacteria [20]. Then whether rhubarb enema regulates the short-chain fatty acid-producing related intestinal flora, thereby improving the intestinal barrier, reducing intestinal inflammation, and ultimately delaying the progress of CKD, remains to be further explored.

Therefore, this study intends to investigate whether rhubarb enema regulates the microflora related to the production of short-chain fatty acids and increases the level of short-chain fatty acids in the intestines, thereby improving the intestinal mucosal damage of CKD.

## 2. Materials and Methods

### 2.1. Animals

32 male Sprague Dawley rats, 6-8 weeks old, were purchased from Guangdong Medical Experimental Animal Center (Guangzhou, China). They were fed specific pathogen-free food and water and kept under a 12-hour light/dark cycle, then raised at 25°C. All animal studies in this experiment were approved by the Animal Experiment Ethics Committee of Guangdong Provincial Hospital of Traditional Chinese Medicine (Ethical number 2019030).

The article "Rhubarb Enema Increasing Short-Chain Fatty Acids that Improves the Intestinal Barrier Disruption in CKD May Be Related to the Regulation of Gut Dysbiosis" was published in 2022. Journal: Biomed Res Int.

This experiment used 5/6 nephrectomy rats to form a model of chronic renal failure. The specific method refers to our previous research [19]. At the 8th week after modeling, blood was collected from the orbit to determine the blood creatinine level. According to the blood creatinine level, the animals were randomly divided into 3 groups: the model group (5/6 nephrectomy rats without enema), the rhubarb enema group (5/6 nephrectomy rats giving rhubarb enema), and the carbonated sevelamer group (5/6 nephrectomy rats giving carbonated sevelamer enema). Another 8 sham-operated rats served as the sham-operated control group with 8 rats for per group.

### 2.2. Drugs and Reagents

Rhubarb granules were purchased from Jiangyin Tianjiang Pharmaceutical (Jiangsu, China, lot 8w2789); carbonic sevelamer from Sanofi (Paris, France, lot 19051281); and IL-1*β* rat ELISA kit (CSB-E08055r), IL-6 rat ELISA kit (CSB-E04640r), TNF-*α* rat ELISA kit (CSB-E11987r), and IFN-*γ* rat ELISA kit (CSB-E04579r) from Wuhan Huamei Bioengineering Co., Ltd. (Wuhan, China). The H&E staining kit was purchased from Boster Bioengineering Co., Ltd. (Wuhan, China), 2.5% glutaraldehyde electron microscope fixing solution from Biyuntian Biotechnology Co., Ltd. (Shanghai, China), and ZO1 (ab221547), Occludin (ab216327), and Claudin-1 (ab211737) primary antibodies from Abcam (Cambridge, UK). The MagMAX Ultra Microbiome Nucleic Acid Isolation Kit and the Qubit dsDNA HS Assay Kit were purchased from Thermo Fisher Scientific (Massachusetts, USA). All medicines and reagents meet the relevant quality standards.

### 2.3. Preparation of Enema

The concentration of the rhubarb enema used in this experiment was consistent with that of the previous study, wherein 20 g of rhubarb granules is dissolved in 100 ml of double-distilled water and fully dissolved to make 0.2 g/ml rhubarb enema. Carbonated sevelamer, a commonly used intestinal adsorbent in clinic, was used as a positive control drug. According to relevant research, 3 g carbonated sevelamer was dissolved in 100 ml of double-distilled water to make 3% sevelamer enema [21].

### 2.4. Enema Method

Before the rat enema, fasting without water for 12 hours, press the back of the rat to fix it on the frame of the rat, positioning the head and neck behind, the tail and anus in front, the rat's tail facing up, and exposing the anus. Stroked the rat's abdomen to make it defecate and empty the intestine as much as possible. Keep the temperature of the medicine at the same temperature as the rat's rectal temperature (37.5–39°C). Then, insert a straight gavage needle into the rectum of the rat about 6 cm. Pinch the anus and fix the gavage needle, slowly injecting the drug and pinching the anus for about 2 minutes. The enema dose used in this study was 5 ml, once a day, and the total cumulative enema time was 4 weeks. The drugs and instruments were required to be treated aseptically during the enema.

The article "Rhubarb Enema Increasing Short-Chain Fatty Acids that Improves the Intestinal Barrier Disruption in CKD May Be Related to the Regulation of Gut Dysbiosis" was published in 2022. Journal: Biomed Res Int.

### 2.5. Biochemical Analysis

After the animal intervention, 24 h urine was collected in the metabolic cage, centrifuged at 3000 r/min for 10 min in the centrifuge, and the supernatant was taken to obtain a 24 h urine sample; after the animal was anesthetized, blood was collected through the abdominal aorta and placed in the centrifuge for 3000 r/min, centrifuge for 15 min, taking the supernatant and waiting until the serum sample. The urine and serum samples were sent to the laboratory of the Laboratory of Guangdong University Town Hospital, Guangdong Traditional Chinese Medicine Hospital, and the Roche automatic biochemical analyzer (Cobas8000, Tokyo, Japan) was used to detect the urine protein-creatinine ratio, serum creatinine, blood urea nitrogen, and blood uric acid levels.

### 2.6. Enzyme-Linked Immunosorbent Assay

According to the protocol, animal serum is added to the ELISA plate coated with the primary antibody, incubate at room temperature for 1 hour, discard the serum and gradient standard, wash the plate, add the HPR secondary antibody, incubate at room temperature for 45 minutes, and, finally, discard. After washing the plate, add the substrate, incubate at room temperature for 30 minutes, add the reaction stop solution, and immediately measure the OD value in a 450 nm microplate reader, and calculate the result.

### 2.7. Short-Chain Fatty Acid Detection

After the intervention, a sample of animal feces was collected. 50 mg of the sample was weighed, and 400 *μ*l of saturated sodium chloride solution was added to 50 *μ*l of 3 mmol saturated sodium chloride solution, shaking to fully dissolve, and ultrasound testing under low temperature for 1 hour. After sonication, 500 *μ*l ice ether is added, then shake for 10 min to fully extract. At 12000 r/min, 4°C, 10 min, take the supernatant. 0.1 g of anhydrous sodium sulfate is added to the supernatant, shake for 3 min at 4500 r/min, 4°C, centrifuge for 5 min, and take the supernatant for analysis. Take 1 mg/ml SCFAs mixed standard and dilute with ultrapure water to 1 ml.

1, 2, 5, 10, 50, 100, 200, and 500 *μ*g/ml series of working fluids were used. Take 50 *μ*l or more of the working solution. 400 *μ*l of saturated sodium chloride solution is added, and 50 *μ*l of 3 mmol saturated sodium chloride solution is added. Shake to dissolve fully and ultrasound at low temperature for 1 h. The instruments used in this experiment are the GC-MS Agilent 7890B gas phase and the Agilent 5977A MSD mass spectrometer in series. Using SIM mode for detection and MSD ChemStation software for data processing, calculate the absolute content of the target compound in the sample. Chromatographic parameters, Column, Agilent HP-FFAP (25 m +0.32 *μ*m+0.50 mm), injection volume: 2 *μ*l, split ratio: 20 : 1, injection port, 250°C. flow rate, 1.5 ml/min, mass spectrometry parameters, ion source: EI+, Ion source temperature: 280°C, transmission line temperature, 250°C, solvent delay, 3.5 min, scan range, scan 35-200 m/z.

The article "Rhubarb Enema Increasing Short-Chain Fatty Acids that Improves the Intestinal Barrier Disruption in CKD May Be Related to the Regulation of Gut Dysbiosis" was published in 2022. Journal: Biomed Res Int.

### 2.8. Transmission Electron Microscopy of Colon Tissue

The colon tissue was fixed in 2.5% glutaraldehyde solution for 24 hours, dehydrated in gradient alcohol, embedded and solidified, sliced by ultrathin microtome for 60 nm, 3% uranyl acetate-lead citrate double-staining, observed under a transmission electron microscope, and underwent filming.

### 2.9. Histopathology

The kidney and colon tissues were fixed in 10% formalin for 36 hours, dehydrated in an automatic dehydrator, embedded, and then made paraffin specimens, which were cut into 0.3 *μ*m paraffin sections. The paraffin sections were baked at 65°C for 1 h; xylene was deparaffinized and rehydrated in gradient alcohol to water, stained with hematoxylin and eosin solution, then dehydrated in gradient alcohol, transparent in xylene, and covered with a coverslip sheet. After drying, we observe the histological changes under a microscope.

### 2.10. Immunohistochemistry

Bake the paraffin sections of intestinal tissue at 65°C for 1 h, deparaffinize xylene and rehydrate in gradient alcohol to water, remove peroxidase in 3% hydrogen peroxide, wash with PBS, block with 5% BSA for 1 h, add ZO1 (1 : 200), Occludin (1 : 300), Claudin-1(1 : 500) primary antibody, incubate overnight at room temperature, wash with PBS, add HRP secondary antibody, incubate at room temperature for 2 h, wash with PBS, develop color under a DAB microscope, stain with hematoxylin, perform gradient alcohol dehydration, using transparent xylene, mounting with neutral gum. After drying, observe histological changes under a microscope, and use a camera system to take images, and use Image-Pro Plus 6.0 to semiquantitate the positive staining in the image analysis.

### 2.11. Metagenomics Sequencing and Analysis of Intestinal Flora

After the enema intervention, fresh animal feces were collected, and the DNA in the fecal samples was extracted according to the MagMAX Ultra Microbiome Nucleic Acid Isolation Kit instructions. The DNA samples were detected, screened, amplified, and circularized, and a series of DNA circular nanometers were obtained. Balls (DNBs), and the resulting DNBs are added to the mesh holes on the chip using high-density DNA nanochip technology. Sequencing was performed by the combined probe anchored polymerization technology (cPAS). After the sequencing is completed, we will perform follow-up information analysis according to the analysis plan. Use the Biobakery process to perform quality control and comparison annotations on the off-machine sequencing data to obtain species abundance information. The quality control process is mainly carried out through kneaddata, including low-quality sequence filtering and host contamination filtering to obtain high-quality sequences. Further, the high-quality sequences are aligned to the species database through metaphlan to obtain the relative abundance information of the species. Use the vegan program package to calculate the sample alpha diversity (Shannon index) and beta diversity, and use the Bray Curtis distance matrix PCoA graph to show the distance between samples. The permanova method was used to analyze the differences between each index of alpha diversity, and the P value was corrected by multiple tests using FDR. The analysis of species differences between groups is to use the lefse method, with Kruskal-Wallis test P value less than 0.05 and LDA score greater than 2 as the standard to screen out the different species between groups.

The article "Rhubarb Enema Increasing Short-Chain Fatty Acids that Improves the Intestinal Barrier Disruption in CKD May Be Related to the Regulation of Gut Dysbiosis" was published in 2022. Journal: Biomed Res Int.

### 2.12. Correlation Analysis of Intestinal Flora and Disease Phenotype

The association between flora and phenotype is analyzed using Spearman association analysis, and displayed by clustering heat map. Species are the difference species between the groups, and the heat map enrichment group is the species-corresponding enrichment group.

### 2.13. Statistical Methods

SPSS software (version 23.0, IBM Corporation, Almonk, New York, USA) is used for statistical analysis, and the measurement data is used to evaluate whether the data conforms to the normal distribution. Independent samples test is used to compare the data with homogeneous variance between two groups of normal distribution. Multiple sets of data use Single factor analysis of variance. The non-parametric Mann–Whitney test was used to compare non-normally distributed data with heterogeneous variance between the two groups. The non-parametric rank sum test is used to compare rank data between groups. A *p* value of <0.05 was considered statistically significant.

## 3. Results

### 3.1. Rhubarb Enema Significantly Improves the Renal Function of 5/6Nx Rats and Reduces the Level of Systemic Inflammation

There was no significant difference in body weight between the four groups (Figure 1(a)). The baseline blood creatinine level of rats showed no significant difference between the model group, the rhubarb group, and the sevelamer group, which was significantly higher than that of the sham operation group (Figure 1(b)). After 4 weeks rhubarb and sevelamer enema treatment, the blood creatinine and urea nitrogen levels of the model group, rhubarb group, and sevelamer group were significantly higher than those of the sham operation group. The blood creatinine and urea nitrogen levels of the rhubarb enema group were significantly lower than that of the model group (Figure 1(c)). The blood creatinine level of sevelamer enema group was also significantly lower than that of the model group, while the blood urea nitrogen level of the sevelamer group was lower than that of the model group, but no statistical significance between them (Figure 1(d)). The urine protein creatinine ratio of the model group, rhubarb group, and sevelamer group were significantly higher than those of the sham operation group, and the urine protein creatinine ratio of the rhubarb enema group was significantly lower than that of the model group (Figure 1(e)). There was no significant difference in blood uric acid levels among the four groups (Figure 1(f)). In terms of system inflammation indicators, serum IL-1*β*, IL-6, TNF-*α*, and IFN-*γ* levels in the model group, rhubarb group, and sevelamer group were significantly higher than those in the sham operation group. The IL-1*β*, TNF-*α* and IFN-*γ* levels in the rhubarb enema group were significantly lower than that of the model group. The IL-6 level of the rhubarb enema group was lower than that of the model group, but there was no statistical significance. The level of IFN-*γ* in the sevelamer group was significantly lower than that of the model group. The levels of IL-1*β*, IL-6 and TNF-*α* in the sevelamer group had a decreasing trend compared with the model group, but there was no statistical significance. In terms of blood lipids, there was no significant significance in triglycerides among the sham operation group, the model group, and the sevelamer group. The triglyceride level in the rhubarb group was significantly higher than the other three groups, and there was no significant significance in total cholesterol among the four groups (Figures 1(g)–1(l)).

The article "Rhubarb Enema Increasing Short-Chain Fatty Acids that Improves the Intestinal Barrier Disruption in CKD May Be Related to the Regulation of Gut Dysbiosis" was published in 2022. Journal: Biomed Res Int.

### 3.2. Rhubarb Enema Improves Kidney Pathology

Compared with the sham operation group, the kidney of the model group, rhubarb group, and sevelamer group had different degrees of renal tubule brush margin shedding and atrophy, a large number of mononuclear lymphocytes infiltration in tubulointerstitium, and tubulointerstitial fibrosis. However, the above-mentioned lesions in the rhubarb group and the sevelamer group were lighter than the model group (Figure 2).

### 3.3. Rhubarb Enema Increases Intestinal SCFAs

The butanoic acid level of rats in the model group was significantly lower than that of the sham operation group. Compared with the model group, the rhubarb enema group and the sevelamer group could significantly increase the butanoic acid level (Figure 3(a)). Compared with the sham operation group, isobutyric acid has a slight downward trend in the model group, but the isobutyric acid level after rhubarb enema treatment is significantly higher than that of the model group, and the isobutyric acid level in the sevelamer group has an upward trend compared with the model group, but there is no statistical significance between them (Figure 3(b)). The levels of valeric acid and isovaleric acid in the model group were slightly lower than those of the sham operation, but no statistical significance. The levels of valeric acid and isovaleric acid in the rhubarb enema group were significantly higher than those in the model group, but there was no statistical significance between them (Figures 3(c) and 3(d)). The levels of hexanoic acid in the model group were significantly lower than those of the sham operation group, while it was significantly increased after rhubarb enema treatment. The levels of hexanoic acid in the sevelamer group were increased, but there was no statistical significance when compared with model group (Figure 3(e)). The acetic acid and caproic acid were increased in the model group, rhubarb enema group, and sevelamer group, but they were significantly higher than those in the sham operation group (Figure 3(f)). The propionic acid in model group, the rhubarb enema group, and the sham group was significantly lower than that of the sham operation group, and the propionic acid level of the rhubarb group was significantly lower than that of the model group, while the propionic acid level of the sevelamer group was higher than the model group, but it was still significantly lower than the sham operation group (Figure 3(g)).

### 3.4. Rhubarb Enema Improves Intestinal Mucosal Injury in 5/6Nx Model Rats

The height of intestinal villi in the model group, rhubarb group, and sevelamer group was lower than that of the sham operation group, and the intestinal mucosa was edema with local mononuclear lymphocyte infiltration. The rhubarb group and sevelamer enema can improve intestinal mucosal inflammation and edema. State, increase the height of intestinal mucosal villi. The electron microscope results showed that the colon of the sham operation group showed abundant microvilli on the surface of epithelial cells, tight junctions and desmosomes were seen between the cells, and no obvious abnormalities in the structure of mitochondria, while in the model group, the microvilli on the surface of epithelial cells were partially missing, and the epithelial cells were cytoplasmic. Cavitation, tight junctions between cells, no desmosomes, swelling of mitochondrial structure, repair of microvilli on the surface of epithelial cells after rhubarb and sevelamer enema, tight junctions and desmosomes between cells, mitochondrial structure is normal (Figure 4).

The article "Rhubarb Enema Increasing Short-Chain Fatty Acids that Improves the Intestinal Barrier Disruption in CKD May Be Related to the Regulation of Gut Dysbiosis" was published in 2022. Journal: Biomed Res Int.

### 3.5. Rhubarb Enema Increases the Expression of Tight Junction Protein in the Intestine of 5/6Nx Model Rats

The expression levels of intestinal tight junction proteins ZO1, Occludin, and Claudin-1 of rats in the model group, rhubarb group, and sevelamer group were significantly lower than those of sham operation, while the expression levels of ZO1 and Occludin in the rhubarb group and sevelamer group were significantly higher than those in the model. The Claudin-1 expression level in the sevelamer group was higher than that in the model group, but there was no statistical difference (Figure 5).

### 3.6. Rhubarb Enema Regulates Gut Microbiota in 5/6Nx Model Rats

Based on the results of metagenomics sequencing analysis of animal intestinal flora, we can see that there is no significant difference in the diversity or uniformity of the intestinal flora of rats in the sham operation, model group, rhubarb group, and sevelamer group. In terms of relative abundance, the four groups of intestinal flora have different species composition. The specific differential flora was as follow, the bacteria enriched in the sham operation group are *fuscicatenibacter-saccharivorans*. The bacteria enriched in the model group are *methanobrevibacter-smithii*, *bacteroides-uniformis*, *bacteroides-vulgatus*, *desulfovibrio-piger*, *bacteroides-dorei*, *streptococcus- azizii*, *bacteroides-massilliensis*, *desulfovibrionaceae-bacterium*, the bacteria that enriched in the rhubarb group are *helicobacter-japonicus*, *akkermansia-muciniphila*, *parabacteroides-goldsteinii*, *paraprevotella-xylaniphila*, *lactobacillus-spray-acid-sophilin*, *testinihobacterium-minisiella-G3-2012*, *bifidobacterium-animalis*, *bifidobacterium-pseudolongum*, *bacteroides-caccae*, *faecalibaculum-rodentium*, *escherichia-coli*, *bacteroides-faecichinchillae*, *parasutterella-excrementihominis*, *parabacteroides-merdae* (Figure 6).

### 3.7. Correlation Analysis of Intestinal Flora and Disease Phenotype

*Bacteroides-dorei*, *bacteroides-caccae*, and *desulfovibro-piger* enriched in the model group are positively correlated with IL-1*β*, IL-6, TNF-*α*, IFN-*γ*, Cr, BUN, acetic acid, and propionic acid, and are closely related to the intestinal tract connexin Occludin is negatively correlated. *Bacteroides-vulgatus*, *methanobrevibacter-smithii* are negatively correlated with butyric acid, isobutyric acid, valeric acid, and isovaleric acid. *Escherichia-coli* are positively correlated with IL-1*β*, TNF-*α*, Cr, BUN, but negatively correlated with intestinal tight junction proteins ZO1, Occludin, and Claudin-1. *Lactobacillus-acidophilus*, *paraprevotella-xylaniphila*, *helicobacter-japonicus*, *anaerotruncus-sp*, *testinihobacterium-minisiella-G3-2012,* which are enriched in rhubarb, which were positively correlated with butyric acid, isobutyric acid, valeric acid, and isovaleric acid, and negatively correlated with uric acid and caproic acid (Figure 7).

The article "Rhubarb Enema Increasing Short-Chain Fatty Acids that Improves the Intestinal Barrier Disruption in CKD May Be Related to the Regulation of Gut Dysbiosis" was published in 2022. Journal: Biomed Res Int.

## 4. Discussion

Rhubarb is the dried root and rhizome of Rheum palmatum L, R.tanguticum Maxim.ex Balf, or medicinal Rhubarb R.officinale Baill. Studies have shown that rhubarb has a wide range of pharmacological effects such as purgation, diuresis, anti-inflammatory, and anti-oxidation, and it is particularly widely used in protecting the intestinal barrier. Studies by Bajic et al. have shown that rhubarb extract can effectively reduce the level of myeloperoxidase, repair the thickness of the intestinal mucosa, thereby improving 5-fluorouracil-induced intestinal mucosal inflammation [22]. In addition, rhubarb has been used to treat chronic renal failure for a long history. It has a definite effect in reducing the levels of CKD creatinine and urea and delaying the progression of CKD [15].

Enema therapy is a traditional Chinese medicine characteristic therapy, which was first recorded in *shang han lun* by Zhang Zhongjing in the han dynasty. In modern times, enema therapy has been applied to the treatment of various diseases such as uremia, paralytic intestinal obstruction and ulcerative colitis [23]. Practice has proved that enema therapy can not only treat local diseases of the colon and rectum, but also treat systemic diseases [24]. Enema is simple to operate, fast in absorption, and effective, and it can also avoid the adverse irritation of certain drugs to the gastric mucosa.

The intestinal barrier can be divided into intestinal mucosal epithelium, intestinal mucus, intestinal flora, secretory immunoglobulin, intestinal-associated lymphoid tissue, bile salts, hormones, and gastric acid, among which the intestinal mucosal epithelial cells and the tightness between epithelial cells. The mechanical barrier formed by the connection is the most important, which can separate the substances in the intestinal cavity and prevent pathogenic antigens from invading the body [25]. In recent years, the relationship between intestinal flora-intestinal barrier-nephropathy has been gradually clarified, and the intestinal-renal axis theory has been proposed. CKD is accompanied by intestinal flora disorders, urinary toxins derived from intestinal flora increase, and its metabolism. The metabolism also changes significantly: the intestinal barrier structure changes, the barrier function decreases, and the intestinal flora and its metabolites enter the submucosa through the damaged intestinal barrier, inducing systemic inflammation and aggravating the progression of kidney disease [2]. The intestinal barrier is an intermediate link between the upstream intestinal flora and kidney disease, and it is also a key link in the prevention and treatment of CKD. Studies have found that improving the intestinal barrier can effectively delay the progression of kidney disease [26]. Our previous research found that rhubarb enema increases the expression of intestinal connexin, down-regulates the mucosal inflammatory response mediated by TLR4-MyD88-NF-*κ*B in the intestine, improves the intestinal barrier, reduces serum IL-1B and IL6 levels, and reduces renal fiber. The mechanism is related to rhubarb enema regulating the intestinal flora of CKD rats. Emodin enema has a similar effect. It can be seen that the target of rhubarb enema in the treatment of chronic kidney disease is consistent with the theory of intestinal-renal axis [20]. This study once again verified that rhubarb enema can improve the intestinal barrier damage of CKD rats, and that rhubarb enema can increase the level of short-chain fatty acids in the intestine.

The article "Rhubarb Enema Increasing Short-Chain Fatty Acids that Improves the Intestinal Barrier Disruption in CKD May Be Related to the Regulation of Gut Dysbiosis" was published in 2022. Journal: Biomed Res Int.

Disturbance of intestinal flora is the initial link of the gut-kidney axis. Recent studies have shown that intestinal flora disorder is closely related to the occurrence and development of kidney disease. A study suggests that there are differences in the gut microbiota between CKD patients and healthy controls. Specifically, compared with healthy controls, *escherichia-shigella*, *parabacteroides*, *roseburia*, *rectal_group*, *ruminococcaceae_NK4A214_group*, *prevotellaceae_UCG.001*, *hungatella*, *intestinimonas* and *pyramidobacter* were significantly increased in CKD patients. Functional analysis also showed that these bacteria are involved in fatty acid and inositol phosphate metabolism [27]. Another study showed that chronic kidney disease is closely related to the following 9 bacteria, such as *escherichia*-*higella*, *diastria*, *spirulina ND3007 group*, *pseudosyringae*, *rosemary*, *paracoccus*, *clostridium lanceolata*, *collinsella stercoris*, and *bacteroides eggerthii*. These bacterial genera are highly correlated with the levels of indoxyl sulfate and p-cresol sulfate in CKD patients. Predictions of the functional capabilities of these microbial communities indicate that these bacteria are involved in the metabolism of aromatic amino acids (phenylalanine, tyrosine, and tryptophan) [28]. To sum up, the influence of flora disorder on kidney disease is mostly related to changes in flora metabolites, which have a harmful effect on the body.

Short-chain fatty acids are derived from the breakdown of dietary fiber in the intestine by intestinal bacteria. Short-chain fatty acids can provide a large amount of energy for the intestinal epithelium and play an important role in maintaining the intestinal barrier function. So which flora can produce short-chain fatty acids? Research by Zhuang et al. showed that Lactobacillus, the Bacteroidales S24-7 group, and Ruminococcaceae can produce short-chain fatty acids, the abundance of which increases as the proportion of dietary fiber in the diet increases [29]. Ara et al. used metagenomics technology to analyze the flora that can produce short-chain fatty acids. They found that Bifidobacterium spp., Blautia hydrogenotrophica, Prevotella spp., Streptococcus spp., and Bifidobacterium spp. can produce acetic acid [5]. Studies have found that *dalister succinatiphilus*, *eubacterium spp*., *megasphaera elsdenii*, *phascolarctobacterium succinatutens*, *roseburia spp.*, *salmonella spp*., *veillonella spp*., *lactobacillus rhamnosus GG*, and *lactobacillus rhamnosus spp*. can produce propionic acid [30]. Other studies have shown that *anaerostipes spp.*, *coprococcus comes*, *coprococcuseutactus*, *clostridium symbiosum*, *eubacterium rectale*, *eubacterium hallii*, *faecalibacterium spp*., and *roseburia spp*. can produce butyric acid [31]. *Akkermansia muciniphila*, *bacteroides spp*., produces both acetic acid and propionic acid [30]. *Coprococcus spp*., *Roseburia inulinivorans*, *Lactobacillus salcinius JCM 1230*, *Lactobacillus agilis JCM 1048* produces both propionic acid and butyric acid [32].

It can be seen that rhubarb enema may increase the abundance of *akkermansia-muciniphila*, *lactobacillus-acidophilus*, *bacteroides-caccae*, and *faecalibaculum-rodentium* in the intestine of CKD rats, thereby increasing the levels of propionic acid and butyric acid and, ultimately, increasing the intestinal tract barrier connexin to improve the intestinal barrier.

## 5. Conclusion

Rhubarb enema increases the short-chain fatty acid-producing flora in the intestine of CKD rats, such as *akkermansia-muciniphila*, *lactobacillus-acidophilus*, *bacteroides-caccae*, and *faecalibaculum-rodentium*, thereby increasing the levels of propionic acid and butyric acid and, ultimately, increasing the intestinal barrier. Connexin can improve the intestinal barrier, thereby reducing the translocation of intestinal flora and intestinal toxins to the intestinal mucosa and intestinal inflammation, ultimately reducing renal interstitial fibrosis and delaying the progression of CKD.

The article "Rhubarb Enema Increasing Short-Chain Fatty Acids that Improves the Intestinal Barrier Disruption in CKD May Be Related to the Regulation of Gut Dysbiosis" was published in 2022. Journal: Biomed Res Int.

## Figures and Tables

**Figure 1:** General clinical situation after enema: (a) body weight of rats after enema, (b) the level of creatinine before enema in rats 8 weeks after modeling, (c) blood urea nitrogen (BUN) levels after enema in rats, (d) serum creatinine level after enema in rats, (e) urinary protein-creatinine (PCR) ratio after enema in rats, (f) blood uric acid (UA) level after enema in rats, (g) serum IL-1*β* levels after enema in rats, (h) serum IL-6 levels after enema in rats, (i) serum TNF-*α* levels after enema in rats, (j) serum IFN-*γ* levels after enema in rats, (k) serum total cholesterol (TC) level after enema in rats, and (l) serum triglyceride (TG) levels after enema in rats. ∗ vs sham, # vs model.

**Figure 2:** H&E staining of rat kidney tissue after enema (200×).

**Figure 3:** The level of short-chain fatty acids (SCFAs) in the feces of rats after enema: (a) the level of butyric acid in the feces of rats after enema, (b) isobutyric acid level in feces of rats after enema, (c) valeric acid levels in feces of rats after enema, (d) isovaleric acid levels in feces of rats after enema, (e) the level of hexanoic acid in feces of rats after enema, (f) the level of acetic acid in feces of rats after enema, and (g) the level of propanoic acid in feces of rats after enema. ∗ vs sham, # vs model.

**Figure 4:** Intestinal histopathology: (a) H&E staining of rat intestinal tissue after enema (200×) and (b) scanning electron microscope of rat intestinal tissue after enema (30000×).

**Figure 5:** Immunohistochemistry of intestinal paraffin tissue in rats after rhubarb enema. Expression of ZO1, Occludin, Aclaudin-1 proteins in intestinal tissue of rats after rhubarb enema. ∗ vs sham, # vs model.

**Figure 6:** Gut microbiota after rhubarb enema: (a) Shannon index after rhubarb enema of gut microbiota, (b) PCA analysis of gut microbiota after rhubarb enema, (c) relative abundance of gut microbiota after rhubarb enema, and (d) differential gut microbiota analysis after rhubarb enema.

**Figure 7:** Correlation analysis between differential gut microbiota and general clinical indicators and intestinal tight junction proteins.

The article "Rhubarb Enema Increasing Short-Chain Fatty Acids that Improves the Intestinal Barrier Disruption in CKD May Be Related to the Regulation of Gut Dysbiosis" was published in 2022. Journal: Biomed Res Int.

## Data Availability

The data generated for this study can be found in NCBI using accession number PRJNA593972. Other data are also available.
